RETRACTED

# Correlation of Nursing Quality and Complications in the Hemodialysis Room as well as Nursing Countermeasures

**DOI:** 10.1155/2022/1841454

**Published:** 2022-04-04

**Authors:** Hongyan Zhao, Changmin Su

**Affiliations:** Department of Blood Purification Center, The First People's Hospital of Lianyungang, No. 6 Zhenhua East Road, Lianyungang, Jiangsu 222000, China

## Abstract

**Objective:**

This study was designed to analyze the correlation between the nursing quality and complications in the hemodialysis room and to explore the nursing countermeasures to reduce the occurrence of complications.

**Methods:**

A total of 242 patients with renal failure were enrolled in our hospital from May 2020 to May 2021. The complications of the patients within 3 months of hemodialysis treatment were observed and recorded. The nursing quality of the corresponding nurses was evaluated by patients. The correlation between nursing quality and complications in the hemodialysis room was analyzed, and the targeted nursing countermeasures were explored.

**Results:**

Within 3 months of hemodialysis treatment, 69 of the 242 patients with renal failure in this study developed complications, with a complication rate of 28.51% (69/242). There were 33 cases (13.64%) of hypertension, 25 cases (10.33%) of hypotension, 15 cases (6.20%) of imbalance syndrome, and 12 cases (4.96%) of arrhythmia, of which 16 cases (6.61%) had two complications. The service quality of patients with hypertension, hypotension, and arrhythmia was significantly lower than that of patients without these complications (*P* < 0.05). The proportion of low-quality nursing patients with hypertension, hypotension, and arrhythmia was higher than that of patients without these complications (*P* < 0.05). Logistic regression analysis showed that hypertension, hypotension, and arrhythmia in complications in the hemodialysis room were related to the nursing quality (OR > 0, *P* < 0.05).

**Conclusion:**

The risk of complications in the hemodialysis room is high. Among which hypertension, hypotension, and arrhythmia are common and are related to the nursing quality. Nursing countermeasures should be taken to reduce complications in the hemodialysis room.

## 1. Introduction

Hemodialysis is suitable for patients with renal injury and renal failure and is an important way to treat renal failure. It can drain the blood in the body through the dialyser and exchange substances to remove metabolic wastes, achieving the effects of kidney replacement therapy, which is beneficial to maintaining the homeostasis of the body [1]. At present, hemodialysis has been widely used for patients with renal diseases [2]. However, hemodialysis requires highly specialized equipment and has a high risk, which can easily lead to complications such as imbalance syndrome and arrhythmia [3]. Moreover, patients generally do not have enough knowledge on hemodialysis treatment, which may affect treatment compliance, thereby causing complications, reducing the efficacy of hemodialysis treatment, and adversely affecting prognosis [4]. The prevention and treatment of complications in the hemodialysis room are important to improve the prognosis of patients. At the same time, the nursing work in the hemodialysis room is difficult, and professional knowledge and skills are required [5]. It is important that nurses caring for the patients with renal failure patients should have good knowledge and skills about catheter care, use, and management [6]. Professional nursing strategies can decrease complications, prolong service time, and improve life quality for renal failure patients undergoing maintenance hemodialysis treatment [7]. Therefore, it is important to perform high-quality nursing to effectively prevent and control complications in the hemodialysis room, which can reduce the risk of hemodialysis treatment. Based on this, this study analyzed the correlation between the nursing quality and complications in the hemodialysis room and explored the nursing countermeasures to reduce the occurrence of complications, so as to provide a reference for the subsequent risk reduction of complications in the hemodialysis room.

RETRACTED

## 2. Materials and Methods

### 2.1. General Data

After review and approval by the medical ethics committee of the First People's Hospital of Lianyungang, 242 patients with renal failure in the hemodialysis room of the First People's Hospital of Lianyungang (approval number: AF/ZZ-LLWYH-04/01.0) were enrolled from May 2020 to May 2021. Both patients and their families had signed the consent forms. Among them, there were 137 males and 105 females who were aged 32–75 years, with an average age of 46.55 ± 5.43 years. The course of renal failure was 2–7 years, with an average course of 4.43 ± 0.73 years. Eighty one cases had diabetic nephropathy, 85 cases had chronic glomerulonephritis, 40 cases had hypertensive renal damage, and 36 cases had other primary diseases.

### 2.2. Selection Standard

Inclusion criteria were listed as follows: (1) meet the diagnostic criteria for renal failure based on KDOQI Clinical Practice Guideline for Hemodialysis Adequacy: 2015 update [8], (2) maintenance hemodialysis >3 months, (3) normal immune and blood system functions, and (4) normal cognitive function and communication ability as well as competence of the scale evaluation. Exclusion criteria were listed as follows: (1) complicated with malignant tumors, (2) complicated with severe infections, (3) receive other blood purification methods in the last month, (4) receive immunosuppressive agents in the last month, and (5) receive kidney transplantation.

RETRACTED

### 2.3. Nursing Quality Assessment

According to five attributes, tangibility, reliability, responsiveness, assurance, and empathy, of the Servqual scale [9], we designed a nursing quality assessment scale including 22 indicators and 2 major parts using the Delphi method according to the characteristics of the hemodialysis room. Each item in the perception part was rated from “not needed” to “very needed” as 1-5 points, and each item in the expectation part was rated from “not achieved” to “fully achieved” as 1–5 points. The higher score represents the higher perception/expectation of the nursing quality. The overall Cronbach's *α* coefficient of the scale was 0.934, and the test-retest reliability was 0.946 through presurvey and reliability and validity tests. After the patients completed the scale assessment, the service quality (SQ) was calculated as follows: SQ = perceived value-expected value. SQ ≥ 0 indicated high nursing quality (patients were satisfied with nursing quality), and SQ < 0 indicated low nursing quality (patients were dissatisfied with nursing quality).

### 2.4. Complication Assessment

Within 3 months of hemodialysis treatment, hypertension (mean arterial pressure increased by more than 10 mmHg), hypotension (mean arterial pressure decreased by more than 30 mmHg or systolic blood pressure fell below 90 mmHg), imbalance syndrome (neurological syndrome related to dialysis, manifested as headache, nausea and vomiting, and muscle twitching), arrhythmia (confirmed by electrocardiogram), and other complications were recorded.

### 2.5. Statistical Analysis

SPSS 22.0 software was used for data processing. Count data were expressed as percentages and analyzed using *χ*2 test. Measurement data were analyzed by Shapiro–Wilk normality test. Measurement data with normal distribution were expressed as $\bar{x}$ ± *s*, and difference comparison between groups was performed using independent sample *t* test. Measurement data with skewed distribution were expressed as median (quartile spacing) [M (P25, P75)], and difference comparison between groups was performed using Mann–Whitney *U* test. Logistic regression analysis was used to assess the relationship between nursing quality and complications in the hemodialysis room. *P* < 0.05 was considered statistically significant.

## 3. Results

### 3.1. Complications in the Hemodialysis Room

Within 3 months of hemodialysis treatment, 69 of the 242 patients with renal failure in this study developed complications, with a complication rate of 28.51% (69/242). There were 33 cases (13.64%) of hypertension (including hypertension complicated with arrhythmia), 25 cases (10.33%) of hypotension, 15 cases (6.20%) of imbalance syndrome, and 12 cases (4.96%) of arrhythmia, of which 16 cases (6.61%) had two complications (Table 1).

RETRACTED

### 3.2. Comparison of General Data of Patients with and without Complications in the Hemodialysis Room

There was no significant difference in the general data between the two groups (*P* > 0.05), as shown in Table 2.

### 3.3. Correlation Analysis between Nursing Quality and Complications in the Hemodialysis Room

The SQ of patients with hypertension, hypotension, and arrhythmia was lower than that of patients without these complications, and the difference was statistically significant (*P* < 0.05), as shown in Table 3. The proportion of low-quality nursing patients with hypertension, hypotension, and arrhythmia was higher than that of patients without these complications, and the difference was statistically significant (*P* < 0.05), as shown in Table 4. Using nursing quality (1 = low nursing quality and 0 = high nursing quality) as the independent variable and hypertension (1 = yes, 0 = no), hypotension (1 = yes, 0 = no) imbalance syndrome (1 = yes, 0 = no), and arrhythmia (1 = yes, 0 = no) as the dependent variables, the logistic regression analysis showed that hypertension, hypotension, and arrhythmia in the hemodialysis room were related to the nursing quality (OR > 0, *P* < 0.05), as shown in Table 5.

## 4. Discussion

Hemodialysis can effectively remove toxins in the blood and correct electrolyte imbalance, which is the main treatment method for patients with renal failure and an important treatment method to maintain the life of patients [10]. However, the poor physical condition of patients, combined with the need for long-term maintenance of hemodialysis treatment, often leads to complications in the hemodialysis room, which may cause the suspension of hemodialysis treatment and even affect the survival of patients [11]. Therefore, it is important to understand the relevant factors of complications in the hemodialysis room and to actively take measures for prevention and treatment, which is of positive significance for improving the prognosis of patients with renal failure.

The results of this study showed that 69 of the 242 renal failure patients developed complications, with a complication rate of 28.51% (69/242). It was suggested that the risk of complications in the hemodialysis room was high, and thus, it is necessary to analyze the related factors. Moreover, the operation of hemodialysis is complicated, and the nursing staff are required to have high operating skills and emergency handling capabilities. These findings suggested that the relatively high nursing quality in the hemodialysis room is needed, and the low nursing quality may affect the risk of complications in the hemodialysis room [12, 13].

RETRACTED

Hemodialysis hypertension, the most common complication in the hemodialysis room, often causes the mean arterial pressure of patients to increase by more than 10 mmHg. Its continuous development will reduce cardiac function and increase the risk of cerebrovascular accidents, and active prevention should be made [14]. Hemodialysis hypertension generally occurs on the basis of the original hypertension. The dialysis process may remove the antihypertensive drugs and thereby reduce their effects. The high calcium ion concentration in the dialysate causes an aggravation of the condition. Moreover, volume overload due to sodium retention can increase dry weight and cause hypertension [15]. This study confirmed that the nursing quality was related to the occurrence of hemodialysis hypertension in patients with renal failure. It may be due to the fact that nursing staff with high nursing quality focus on helping patients understand their dry weight and instructing patients to adjust their dry weight, thereby controlling blood pressure. Nursing staff with low nursing quality do not pay attention to the specific conditions of patients to make recommendations, resulting in high dry weight of patients and causing hypertension [16]. Nursing staff with low nursing quality may have insufficient nursing experience and fail to choose a reasonable dialysate, which causes patients to be affected by high-concentration calcium ions during dialysis, resulting in increased blood pressure. For hypertension, it is suggested that health education should be strengthened during nursing to help patients adjust their diet, limit intake of water and salt, control dry weight, and pay attention to the calcium ion concentration in the dialysate.

Hypotension is also a common complication in the hemodialysis room, which causes not only discomfort to the patients but also vascular occlusion, affecting the prognosis of the patients [17]. The occurrence of hemodialysis hypotension is closely related to excessive dehydration and excessive ultrafiltration during dialysis [18]. The results of this study showed that the nursing quality was associated with the occurrence of hemodialysis hypotension. It may be due to the fact that nursing staff with low nursing quality fail to adjust the ultrafiltration volume according to the specific situation of the patients, resulting in excessive ultrafiltration volume, even exceeding the cardiovascular compensation, thereby reducing the effective circulating blood volume, and increasing the risk of hypotension occurrence. Moreover, the low nursing quality may cause the ignorance of signs of hypotension such as sweating and dizziness, and the blood volume of patients is not replenished in time, resulting in the occurrence of hypotension [19]. Therefore, during the nursing work in the hemodialysis room, nursing staff should take reasonable measures to prevent hypotension, such as controlling the dehydration speed, adjusting the amount of dehydration, and avoiding excessive dehydration [20]. At the same time, it is possible to control the growth rate of dry weight during dialysis by correctly assessing the patients' dry weight [21]. During dialysis, the vital signs of patients should be carefully observed, and replenishing blood volume should be conducted in time to reduce the occurrence of hypotension. In addition, the use of antihypertensive drugs can be reduced to prevent hypotension in patients at higher risk for hypotension [22].

RETRACTED

The occurrence of arrhythmias in the hemodialysis room is closely related to the development of heart diseases such as pericarditis and metabolic cardiomyopathy, the accumulation of substances, excessive body fluids, and electrolyte disturbances [23, 24]. This study demonstrated that the occurrence of arrhythmias in the hemodialysis room was also related to the nursing quality, which may be due to the fact that the nursing staff with low nursing quality are relatively insensitive to the changes of the vital signs of patients and fail to notice the arrhythmia precursor in time [25]. Nursing staff with low nursing quality fail to relieve negative emotions such as tension and anxiety, resulting in the increased stress response of patients, leading to the increased pulse rate or irregular pulse, and thereby increasing the risk of arrhythmia occurrence. Therefore, in the process of dialysis treatment, the nursing staff should carefully focus on the changes of vital signs and respond in time [26]. For patients with preexisting heart diseases, symptoms should be actively controlled prior to dialysis treatment [27].

A limitation of this study needs to be stated. Since only 242 patients were enrolled, the effects of nursing quality on complications of renal failure patients in the hemodialysis room require to be investigated in a larger sample size.

## 5. Conclusion

The risk of complications in the hemodialysis room is high. Among which hypertension, hypotension, and arrhythmia are common and are all related to the nursing quality. Nursing measures should be taken to reduce complications in the hemodialysis room.

RETRACTED

## Figures and Tables

**Table 1:** Complication rates of patients.

Complications	Cases	Total	Cases of two complications
Hypertension	33 (13.64%)	69/242 (28.51%)	16 (6.61%)
Hypotension	25 (10.33%)		
Imbalance syndrome	15 (6.20%)		
Arrhythmia	12 (4.96%)		

**Table 2:** General data of patients with and without complications in the hemodialysis room.

Data		Complication group (*n* = 69)	No complication group (*n* = 173)	Statistical value	*P*
Gender [*n* (%)]	Male	41 (59.42)	96 (55.49)	*χ*2 = 0.310	0.578
	Female	28 (40.58)	77 (44.51)		

Age ($\bar{x}$ ± *s*, year)		46.84 ± 4.56	46.43 ± 5.75	*t* = 0.533	0.595

Course of renal failure ($\bar{x}$ ± *s*, year)		4.45 ± 0.65	4.42 ± 0.75	*t* = 0.319	0.750

Primary diseases [*n* (%)]	Diabetic nephropathy	21 (30.43)	60 (34.68)	*χ*2 = 1.309	0.727
	Chronic glomerulonephritis	24 (34.78)	61 (35.26)		
	Hypertensive kidney damage	11 (15.94)	29 (16.76)		
	Others	13 (18.84)	23 (13.29)		

**Table 3:** Nursing quality of patients with and without complications in the hemodialysis room.

Complications		SQ [M (P25, P75)]	U	*P*
Hypertension	Yes	−2.00 (−3.00, −1.00)	5.292	<0.001
	No	1.00 (−2.00, 4.00)		

Hypotension	Yes	−4.00 (−4.00, −3.00)	6.534	<0.001
	No	1.00 (−1.00, 3.00)		

Imbalance syndrome	Yes	0.00 (0.00, 1.50)	0.065	0.948
	No	1.00 (−2.00, 3.00)		

Arrhythmia	Yes	−2.50 (−4.00, −0.50)	3.500	<0.001
	No	1.00 (−2.00, 3.00)		

**Table 4:** Relationship between complications in the hemodialysis room and nursing quality.

Complications	Low nursing quality	High nursing quality	*χ*2	*P*
Hypertension (*n* = 33)	27 (81.82)	6 (18.18)	29.707	<0.001
Hypotension (*n* = 25)	23 (92.00)	2 (8.00)	33.163	<0.001
Imbalance syndrome (*n* = 15)	3 (20.00)	12 (80.00)	2.390	0.122
Arrhythmia (*n* = 12)	9 (75.00)	3 (25.00)	6.949	0.008

**Table 5:** Logistic regression analysis results of the correlation between nursing quality and complications in the hemodialysis room.

Complications	Factor	B	SE	WaId	*P*	OR	95% CI
Hypertension	Nursing quality	2.255	0.475	22.537	<0.001	9.537	3.759–24.198
Hypotension	Nursing quality	3.163	0.751	17.729	<0.001	23.648	5.424–103.105
Arrhythmia	Nursing quality	1.633	0.681	5.756	0.016	5.118	1.348–19.424

## Data Availability

The data that support the findings of this study are available from the corresponding author upon reasonable request.
